The article "Exploring the Study of miR-1301 Inhibiting the Proliferation and Migration of Squamous Cell Carcinoma YD-38 Cells through PI3K/AKT Pathway under Deep Learning Medical Images" was published in 2022. Journal: Comput Intell Neurosci.

# Exploring the Study of miR-1301 Inhibiting the Proliferation and Migration of Squamous Cell Carcinoma YD-38 Cells through PI3K/AKT Pathway under Deep Learning Medical Images

**DOI:** 10.1155/2022/5865640

**Published:** 2022-02-10

**Authors:** Chaofan Gong, Rohit Bhargava, Chandrajit Bajaj

**Affiliations:** ^1^Cancer Center at Illinois, University of Illinois at Urbana-Champaign, Urbana, IL 61801, USA; ^2^Department of Computer Science, Computational Visualization Center, University of Texas at Austin, Austin, TX 78705, USA

## Abstract

With the rapid development and application of deep learning medical image recognition, natural language processing, and other fields, at the same time, deep learning has become the most popular research direction in the field of image processing and recognition. Through deep learning medical image recognition technology, it is of great significance to explore the research of miR-1301. The purpose of this article is to use an improved CNN neural network model algorithm combined to contrast the experimental groups and use deep learning medical imaging technology to study the mechanism by which miR-1301 inhibits the proliferation of carcinoma YD-38 cells through the PI3K/AKT pathway. This paper studies the method of image recognition of squamous cell carcinoma YD-38 cells using a convolutional neural network (CNN). First, a CNN classification model for the characteristics of YD-38 cell images is constructed. Then, pretraining and dropout technology are used to improve and optimize the proposed CNN model to improve the robustness of the model. In this paper, the miR mimic group and the miR blank group and the PI3K/AKT pathway inhibitor Wortmannin were selected to jointly treat YD-38 cells. The expression of mRNA in miR-1301 in HGF-1 was determined using RT-PCR (real and real-time fluorescence and YD-38 cells). The blank plasmids and the miR-1301 mimic (miR-1301 mimic) were transfected into YD-38 cells. The experiments were divided into two groups in the miR-1301 blank group and the miR-1301 simulation groups, respectively. The proliferation capacity of YD-38 cells was prepared in 1.5 ml sterile EP tubes and then diluted with medium for the proliferation of the cells. The scratch test and Transwell test were used to detect the effect of miR-1-3p on the migration and invasion of liver cancer cells. In this paper, CCK-8 experiment, clone formation experiment, flow cytometry, scratch experiment, and Transwell chamber experiment are used to analyze the effects of target gene CAAP1 on the proliferation, apoptosis, migration, and invasion of liver cancer cells. This paper uses CCK-8 to detect five kinds of the effect of miRNA on the proliferation ability of liver cancer cells and the effect of miR-1-3p on the proliferation ability of liver cancer cells. Experimental studies have shown that, compared with the miR blank group, the expression of PI3K and p-AKT was significantly downregulated in the miR mimic group after 24, 48, and 72 hours and the phosphorylation level of AKT was also significantly reduced (*P* < 0.05).

## 1. Introduction

At present, most of the classification and regression algorithms for squamous cell carcinoma YD-38 cell images belong to shallow learning [1, 2]. Express complex functions with fewer parameters achieve a better way of function expression characteristics of data sets from a small number of samples [3, 4]. Therefore, this article attempts to apply deep learning to the image classification and in-depth study of miR-1301 inhibiting. Deep learning is the intrinsic rules and representation hierarchy of learning sample data, and the information obtained during these learning processes is greatly helpful to the interpretation of data such as text, images, and sound. The ultimate goal is to make the present model have more accurate analytical learning ability, to identify data such as text, image, and sound.

In the research of cell value-added and migration based on deep learning medical images, many scholars have studied them and achieved good results. For example, Wang K proposed a CSF (cerebrospinal fluid) reverse image recognition model based on reverse CNN [5]. Choi HS uses deep CNN as a feature extractor to better understand the segmentation of nerve cell membranes, then, uses the random forest method as a classifier, and compares it with mainstream methods to prove the effectiveness of the method [6]. He T combines the artificially designed kernel features with the features learned by CNN, by capturing the color, texture, and shape information of the area around the core, and using CNN to control the type of mitosis and reduce the sensitivity to artificially designed feature boundaries [7]. Gong F uses an improved algorithm based on deep CNN. First, ZCA is used to preprocess the image of abnormal breast cells to reduce the correlation between feature data, thereby reducing the redundancy between the data, and then the deep convergence neural network is used to perform case cell image classification [8].

In this paper, an adaptive convolutional network model of squamous cell carcinoma YD-38 cell image representation and reconstruction algorithm is proposed, and this model is combined with SPM to finally realize image classification. In this paper, the CCK-8 experiment, clone formation experiment, flow cytometry, and Transwell chamber experiment were used to analyze the effect of miR-1301. The present adaptive convolutional network model is an improved neural network model with an iterative shrinkage threshold algorithm that enables faster convergence, higher computational result accuracy, and faster efficiency.

## 2. Method of miR-1301 Based on Deep Learning Medical Images in Inhibiting the Proliferation and Migration of Squamous Cell Carcinoma YD-38 Cells through the PI3K/AKT Pathway

### 2.1. Research Progress on the Relationship between miR and Cancer Cells

#### 2.1.1. Introduction to miRNA

MicroRNA (miRNA) is a small uncoded double-stranded RNA molecule with 20–22 nucleotides that can be expressed in gene conversion. By identifying UTR mRNA3 target genes and combining them with complementary sequences intact or incompletely, they destabilize mRNA and inhibit mRNA translation and regulate gene expression after transcription or transcription [9, 10]. The maturation of miRNA can be split into two. The first is the original miRNA transcript (pri-miRNA) in the nucleus, which is then cut into a precursor miRNA (pre-miRNA) with a hairpin structure of about 70 nt. The second stage is the transfer of pre-miRNA, which is cleaved into a double-stranded RNA of approximately 22 bp by another enzyme. One strand becomes a mature miRNA and participates in regulating gene expression, while the other strand usually degrades rapidly. The phosphate group at the end of mature miRNA and the hydroxyl group at the end are unique markers for RNA fragments of the same length. Certain miRNA subgroups are lean to cells, such as cell proliferation, differentiation, and apoptosis [11]. Although their biological functions are unclear, recent experiments have shown that miRNAs of cancer. The expression level of miRNA in cancer is generally around 20 ng, and the expression specificity in normal cells and cancer cells is that normal cells express specific proteins after differentiation to form tissues or organs with specific functions. In cancer cell protein expression profiles, cancer cells often show some proteins expressed in embryonic cells. Most cancer cells also have a high telomerase activity. In addition, the expression of protein components related to the malignant proliferation and diffusion of cancer cells is often abnormal. The miRNA is encoded by a noncoding single-stranded RNA molecule of about 22 nucleotides, which can effectively participate in posttranscriptional gene expression regulation in plants and plants.

#### 2.1.2. Relationship between miRNA and Cancer

Many studies conducted that genome-wide analysis has determined that the expression levels of miRNA are different. Comparative miRNA expression studies have found that some miRNAs (such as miR-1301) are usually downregulated. These observations indicate that these miRNAs are very important [1, 12]. There have been many studies analyzing the functions of these miRNAs. Further miRNA expression profile analysis studies have shown that miRNA can be used as an indicator of prostate cancer diagnosis and prognosis. Recently, some scholars proved that restoring the expression of miR-1301 in the YD-38 cells of the front row squamous cell carcinoma inhibited cell proliferation, migration, and invasion.

A research shows that whole-genome analysis has shown that the expression levels of miRNAs are different. Comparative miRNA expression studies have found that certain miRNAs (such as miR-1301) are usually reduced [13]. These observations indicate that these miRNAs are very important in these miRNAs. Further studies on the analysis of miRNA expression profiles have shown that miRNA can be used as a marker for the diagnosis. Recently, some researchers have shown that by restoring the expression of miR-1301 in YD-38 cells of first-line during the proliferation and development of cells, different cell carcinomas will invade and be blocked during the migration period. The pathogenesis of miRNAs in tumorigenesis is very clear; that is, miRNAs can act as tumor suppressor genes or oncogenes during tumor development. If miRNAs are upregulated in tumors, they may be oncogenes that negatively regulate tumor suppressor genes and affect cell growth and apoptosis pathways to promote tumorigenesis [14]. These miRNAs are based on the biological functions of target genes, and they regulate them to function as oncogenes or tumor suppressor genes. Mature miRNAs by binding to target mRNA specific (incomplete complementary), leading to its cleavage degradation or translation inhibition, exerts its negative regulation in posttranscriptional gene expression, ensuring the normal progress of cell cycle program and terminal differentiation. Its abnormal gene development can cause changes in mature miRNAs expression, causing variation in cell proliferation and apoptosis, and eventually tumor formation.

miRNA is expected to become a new biological of diseases, and it may also become a target for new cancers. For example, epigenetic changes in miRNAs (such as methylation) can affect the ability of cancer cells to invade and migrate.

#### 2.1.3. Relationship between miR-1 and Cancer

miR-1301 was originally thought to control muscle development and differentiation. However, current research shows that it plays an important role in certain cancers, such as rhabdomyosarcoma, the most common soft tissue sarcoma in children. Studies have shown that miR-1301 is rarely detected in primary rhabdomyosarcoma. The reexpression of miR-1301 in tumor cells oral cavity cells inhibits the growth of squamous cell carcinoma YD-38 cells in xenotransplanted mice [15, 16]. Studies have reported that miR-1 is downregulated in human malignant tumors.

Abnormal expression of miR-1301 in liver cancer, lung cancer, prostate cancer, and rhabdomyosarcoma inhibits tumor cell growth. In cardiomyocytes, miR-1301 regulates cell apoptosis by inhibiting BCL2. In the field of oral cancer research, abnormal expression of miR-1301 induces apoptosis by enhancing the activity of caspases 3 and 7, cleaving polyadenylic acid diphosphate ribose transferase-1 (PARP-1), and depleting antiapoptotic Mcl-1. By targeting LASP1, miR-1301 in oral cancer acts as a cancer suppressor gene [17]. All observations suggest that miR-1301 dysregulation plays a role in the tumor suppressor gene by losing its inhibitory effect on LASP1, IGF-1, IGFR-1, BCL2, and other target genes. In the field of oral cancer research, aberrantly expressed miR-1301 regulates a range of biochemical events causing multiple Mcl-1 cell morphology changes, including altered membrane symmetry, cell shrinkage, nuclear fragmentation, and chromatin condensation, eventually causing apoptosis in Mcl-1 cells.

### 2.2. Tumor Cell Image Recognition Based on ADN and SPM

#### 2.2.1. Building a CNN Model

*(1) Image Preprocessing*. The original YD-38 squamous cell carcinoma is a very large color image. In digital image processing, the image is usually scaled first to reduce the number of subsequent calculations. The grayscale image still reflects all and part of the color, distribution and color characteristics, and brightness level of the entire image. The image preprocessing method of the CNN model is to flip the existing graph, translation, atomization, dedryness, and other methods, increase the sample size, facilitate training, and diversify the training situation, making the obtained results more reliable.

*(2) CNN Structure*. Under normal circumstances, there is usually a lot of information that interferes with the image of YD-38 squamous cell carcinoma. This is mainly caused by two reasons: first, it may be affected by noise during imaging and imaging; second, due to some other cells in the slice (such as inflammatory cell granules) and the morphology of diffuse cells are not different, turbidity is left in the picture of YD-38 squamous cell carcinoma, which is very unfavorable for cell extraction [18]. CNN's unique local receptive field, weight sharing, and subsampling structure features reduce computational complexity while meeting the requirements for rotation, scale, and offset. The convolutional neural network is a multilevel network model. In the field of image processing, its input is the image data composed of multiple channels. After multiple convolution, pooling, and activation in the network, features were extracted. Then, the output through the full connection layer is the forward transmission process of the network.

#### 2.2.2. Inference Feature Map

For a given layer *l*, input image *y*, and filter *f*, the purpose of inference is to find the feature map *z*_*l*_ to minimize the cost function *C*_*l*_ th, and each layer has deconvolution. For this reason, the iterative shrinking threshold algorithm, ISTA, is used (Iterative Shrinkage-Thresholding Algorithm, ISTA) to solve [6]. The gradient iteration framework and contraction step are used in the solution process.

*(1)Gradient Step*. This involves the gradient of the reconstruction term with respect to *z*_*l*_ falling toward *g*_*l*_:

(1) $$\begin{array}{c} g_{l}=R_{l}^{T}\left(R_{l}z_{l}-th\right). \end{array}$$

To calculate this gradient, we use the feature map and filter and the switch settings of the next layer to reconstruct the input *t*^2^ = *R*_*l*_*z*_*l*_ and then calculate the reconstruction error *t*^2^ − *t*. This requires the network to perform feedback propagation through the projection operation (the layer alternately performs convolution (*F*^*T*^*h*) and pooling (*P*_*s*_*h*) and finally generates a gradient *g*_*l*_). With the gradient, you can update *z*_*l*_:

(2) $$\begin{array}{c} z_{l}=z_{l}-\frac{\lambda_{l}}{3_{l}g_{l}}. \end{array}$$

The parameter*/3*_*l*_ is used to set the size of the gradient.

*(2) Shrinking Step*. After the gradient step, a shrinking operation is performed on each element, so that the small element in *z*_*l*_ becomes zero, thereby increasing its sparsity.

*(3) Pooling/Depooling*. Update the switches of the current layer through the pooling operation [*p*_*l*_, *s*_*l*_) = *P*(*z*_*l*_*h*), followed by the depooling operation *z*_*l*_ = *U*_*sl*_*p*_*l*_, which achieves two major functions. (1) When adding layers to the top, ensure that the input can be accurately reconstructed through pooling. (2) The updated switch can reflect the modified feature mapping value. Once the reasoning is confirmed, the switch will also be fixed to prepare for the training of the upper layer. Therefore, another purpose of reasoning is to optimize the switch settings of the current layer. The pooling layer is part of the CNN network, and the pooling method includes maximum pooling and average pooling, that is, maximum feature points within the neighborhood and better texture extraction. Average pooling is only averaging the feature points in the neighborhood and better retaining the background. Depooling is the reverse process, and pooling can reduce features, reduce parameters, and speed up the calculation speed.

*(4) Full Iteration.* The iterative process of a single ISTA includes the above three steps of gradient, shrinkage, and pooling/depooling. In this process, 10 ISTA iterations are performed for each picture of each layer.

Both the reconstruction operation *R* and the projection operation *R*^*T*^ are very fast, including only convolution, summation, and pooling/depooling operations. These operations can be parallelized, which can effectively shorten the running time. Although the gradient step is linear, the whole model is nonlinear, because the sparsity in the shrinking step and the setting of the switch in the reconstruction operation change the result of pooling/nonpooling.

#### 2.2.3. Learning Process

The purpose of learning is to estimate the filter *f* in the model, and all images *Y* = *ot*^*l*^,…, *t*^*i*^, *…*, *t*^*N*^*}* share the filter. For a given layer *l*, calculate *z*^*i*^ through inference. Regarding *f*_*l*_ as 0, the following linear system can be obtained:

(3) $$\begin{array}{c} \left.I_{i=0}^{N}\right)\left.z_{l}^{iT}P_{s_{l-0}}^{iT}R_{l-0}^{iT}\left(t_{l}=I_{i=0}^{N}\right)z_{l}^{iT}P_{s_{l-0}}^{iT}R_{l-0}^{iT}\right]t^{i}. \end{array}$$

Use the conjugate gradient algorithm (conjugate gradients, CG) to solve this linear system. The algorithm of all layers in the learning model has been given in the adaptive deconvolution algorithm, which alternately solves *z*_*l*_ and *f*_*l*_. In each iteration, *z*_*l*_ performs an ISTA inference, and *f*_*l*_ performs two CG iterations, repeating 10 times.

#### 2.2.4. Spatial Pyramid Matching

Suppose there are two point sets *X* and *Y* (each point set is D-dimensional, and the space in which they are located is called a feature space below). Learning principle of the algorithm: if the input image is *M*, the feature map of MI can be obtained through the convolution core and the input image, but there will be a loss in the actual application process. The improved CNN algorithm introduces the loss function to reduce the computational loss. The feature space is divided into different scales 0,…, *L*, and *2*^*y*^ bins are delineated in each dimension of the feature space under the scale *γ*; then, the D-dimensional feature space has a total of *D* = *2*^*y*^ bins.

Let *H*^*y*^ and *H*^*y*^ represent the histograms of *X* and *Y*, respectively, so *H*^*y*^ (*ih*) and *H*^*y*^ (*ih*) are the numbers of points from *X* and *Y* that fall into the *i*-th bin in the grid. Then, the matching degree *b* is calculated by the function:

(4) $$\begin{array}{c} K=H_{X}^{y},H_{Y}^{y}\left(I_{\mathrm{i=0}}^{D}\right.\min\left(H_{X}^{y}\right)i,\left(H_{Y}^{y}\right)\left(ihh\right). \end{array}$$

For the convenience of description, *K* (*H*^*y*^,*H*^*y*^) is abbreviated as *K*^*y*^ below. Since the matching number on the scale *l* includes the matching number of the finer scale *γ* + 1, the final matching number of the scale *l* is equal to *K*^*y*^ − *K*^*y*^ ^+^ ^*o*^, *y* = *t*, *…*, *t* − *o*. The relative weight of the scale *γ* is set to *o*, which is inversely proportional to the width of the scale cell. Intuitively speaking, matching under different scales should be given different weights. Obviously, the weight of the large scale is small, and the weight of the small scale is heavier. In the end, the degree of matching between the two point sets is defined as

(5) $$\begin{array}{c} Y^{t}\left(X,Y\right)=K^{t}+I_{y=t}^{t-o}\frac{o}{2^{t-y}}\left(K^{y}-K^{y+o}h\right.=\frac{o\;K^{t}}{2^{t}}+I_{y=o}^{t}\frac{o}{2^{t-y+o}}K^{y}. \end{array}$$

SPM actually uses the spatial coordinates of the image to replace the aforementioned hypothetical feature space and uses the pyramid construction method to decompose the image space into multiscale bins (squares of different proportions). Then, like BOW Words (BagOF Words, BOW), we build an M-size dictionary so that each function is displayed in a word in the dictionary. The education process of the dictionary is completed in the functional area, and the function used is intensive SIFT; the number of each word in each statistic bin and the matching degree of the last two images are defined as

(6) $$\begin{array}{c} K^{t}X,Y=I^{M}Y^{t}\left(X_{m},Y_{m}h\right). \end{array}$$

When *L* = 0, the model degenerates into BOW.

Calculating the similarity by formula (5), the final classification decision function of SVM can be written as

(7) $$\begin{array}{c} f\left(x\right)=\left(I_{i=o}^{n}a_{i}t_{i}x_{i}h^{T}x+h=I_{t=o}^{n}a_{i}t_{i}<x_{i},xh+h\right). \end{array}$$

Here, *x* is all training samples, *x* is the sample to be classified, and only the corresponding support vector of *α* is greater than 0 (nonsupport vectors are all equal to 0). Rewrite formula (7), and divide the training samples into positive and negative samples:

(8) $$\begin{array}{c} f\left(x\right)=I_{i=o}^{k^{+}}+a_{i}<x_{i},xh-I_{i=o}^{k^{-}}a_{i}<x_{i},xh+h. \end{array}$$

The above types of results are more intuitive. According to the formula, it can be observed that the data on the right is actually the inner product of all positive samples that have not yet been sorted, which is the similarity described in equation (5). SVM can use core functions instead of internal products, and this equation can also be used in equation (5). The core function of the intersection of the equiangular lines replaces the internal product, and the internal product is the core function corresponding to the Euclidean distance. Use chi-square kernel SVM to use SPM in classification problems. The learning process of SVM is the process of learning these parameters *a* and *b*. These parameters weigh each training sample, and heavier training samples are more decisive. Therefore, the classification problem is essentially a problem of matching test samples with training samples. Therefore, SPM can be used to solve classification problems. SVM is able to separate different class samples in the sample space. In other words, given some labeled training books (supervised learning), the SVM algorithm outputs an optimized hyperseparation plane. This time, VS2015 + OpenCV3.4.1 was used to implement the SVM algorithm, complete the training of the dataset, generate the XML files, and then realize the recognition and classification of the pictures by calling the XML files.

## 3. Under Deep Learning Medical Images, Exploring the Experimental Study of miR-1301 Inhibiting the Proliferation and Migration of Squamous Cell Carcinoma YD-38 Cells through the PI3K/AKT Pathway

### 3.1. Experimental Research on Image Recognition of Oral Squamous Cell Carcinoma YD-38 Cells Based on Deep Learning

This paper divides the model into two stages of training. In the first stage, 300 images are randomly selected from the original YD-38 cell database, 100 images per category, a total of 3 categories; the image is divided into blocks in MatLab, and each original 80 × 60 image is divided into four 40 × 30 small images, and finally, 1200 images can be obtained. This article uses the expanded new image data set to train the CNN model. This paper uses an improved CNN model using an iterative shrinkage threshold algorithm to make it more robust. Image segmentation in MatLab: according to the RGB principle, using grayscale, dark gray and white categories represent cancer cells and normal cells, respectively. The original image recognition method is not a perfect identification model, and the recognition effect is not obvious. The image recognition of the improved CNN model method used in this paper has high recognition accuracy and faster recognition efficiency and can obtain experimental results. After the model converges, we save the model parameters. The second stage is the initial squamous cell carcinoma training data set from YD-38. Retrain the model, but use the parameters obtained in the first step to initialize the model parameters, which significantly reduces the model training time and speeds up the convergence of the entire model.

### 3.2. Experimental Materials

Human normal oral epithelial cells HGF-1 and oral squamous cell carcinoma YD-38 were purchased from ATCC cell bank in the United States; TRIzol kit, Prime-ScriptRT kit, fetal bovine serum, RPMI-1640 medium, negative control (miR-NC) or miR-1301 mimic, liposome 2000, and CCK-8 kit were purchased from Addison. Antibodies to PI3K, p-AKT, and AKT were purchased from Santacruz Company. PI3K, p-AKT, AKT, and GAPDH primers were synthesized by Shenggong Bioengineering Company.

### 3.3. Experimental Methods and Data Collection

#### 3.3.1. RT-PCR (Real-Time Fluorescent Quantitative PCR) Measures the mRNA Expression of miR-1301 in HGF-1 and YD-38 Cells

Primers were selected for 15–30 bp in length and did not contain their own complementary sequences, with less than four complementary or homologous bases between the primers. Treatment of negative control: turn on the biological fan to detect dust particles and prevent pollution. In this paper, the miR simulation group and the blank group comparisons are selected, and we optimize the CNN model to improve the robustness and ensure computational effectiveness.

#### 3.3.2. Cell Transfection

The blank plasmid and miR-1301mimics (miR-1301 mimics) were transfected into YD-38 cells.

The following experiments are divided into miR-1301blank and miR-1301mimics2 groups.

*(1) Prepare Solution A and Solution B in Two Sterile 1.5 ml EP Tubes (the Following Is the Amount Used to Transfect Five-Well Cells)*. Solution A to detect the effect of the miR blank group on the proliferation ability of squamous cell carcinoma YD-38 cells: dilute the miR-13011.25 *μ*g plasmid with serum-free medium Opti-MEM, the final volume is 25 *μ*L, gently pipette to mix, and centrifuge briefly. Solution A to detect the effect of miR mimic group and miR blank group on the proliferation ability of YD-38 cells: dilute 0 *μ*g, 0.25 *μ*g, 0.5 *μ*g, 0.75 *μ*g, 1.25 *μ*g, and 1.75 *μ*g with serum-free medium Opti-MEM miR-1301, the final volume is 25 *μ*L, gently pipette to mix, and centrifuge briefly.

Liquid A for detecting the effect of miR-1301 on the proliferation of squamous cell carcinoma YD-38 cells: dilute 1.25 *μ*g plasmid of miR-1301 or 2.5 *μ*L each of miR-1301 with serum-free medium.

Opti-MEM, the final volume is 25 *μ*L, liquid B : Before preparation, mix the liposome Lipofectamine2000 gently, then dilute 1.25 *μ*L Lipofectamine 2000 with Opti-MEM, the final volume is 25 *μ*L, gently pipette to mix, and leave it at room temperature for 5 min. Add liquid B to liquid A, pipette gently 3–4 times, and leave it at room temperature for 15–20 minutes.

*(2) Preparation for Transfection*. When it is about 15–18 minutes, take out the culture plate, aspirate the original culture medium, wash twice with 1 × PBS, aspirate the PBS, and slowly drop 10 *μ*L of the above-mentioned mixed transfection solution into each corresponding well. Then, add 90 *μ*L serum-free Opti-MEM medium to each well, mix well, and incubate at 37°C and 5% CO_2_.

*(3) Change the Medium*. Change the medium 4–6 hours after transfection, aspirate the stock solution, add 100 *μ*L of 10% FBS, nonantibiotic-free DMEM high-glycemic culture medium to each well, and continue to culture in the cell incubator.

After transfection for 24 h, 48 h, and 72 h (when detecting the effect of miR mimic group and miR blank group on the proliferation ability of squamous cell carcinoma YD-38 cells, only the OD value after 48 h of transfection), aspirate the original culture medium, and add 100 *μ*L of complete culture medium and 10 *μ*L of CCK-8 reagent to each well, gently shake the culture plate to mix, and then use a microplate reader to detect the absorbance value (ie OD value) of each well at a wavelength of 450 nm after 3 hours in a 37°C incubator. 0 h is used to determine the initial density of cells.

*(4) Exposure Appraisal*.

  Prepare the dark room: pour the programmer, installation tools, and tap water into the plastic tray for use in the dark room.
  Exposure preparation: after incubating the membrane with the secondary antibody, wash the membrane with TBST, and then add 200 *μ*L of luminescent solution A and B to the centrifuge tube and mix.
  Coat the plastic film with a zipper on the cassette, move the washed PVDF film up to the plastic film, remove the remaining liquid, pour the light liquid evenly on the PVDF film, and then use another layer of foil carefully Cover PVDF.
  Exposure: put the X-ray film in a dark room, cut it into a suitable size with scissors, open the cassette, and then place the X-ray film on the film. After installation, it cannot be moved. Close the cassette, start timing, and adjust the exposure time according to the fluorescence intensity observed by naked eyes, usually 1–5 minutes. Use multiple reports to achieve the best results. After the exposure is completed, open the cassette and take out the X-ray film, immerse it in the programmer solution, and continue to shake it to grow it. After noticing the visible band under the red light (usually about 1 minute), immediately immerse it in the fixing solution (5–10 minutes). The film is transparent. After rinsing off the remaining fixative with tap water, let it dry at room temperature and store the film in a cool and dry place.

*(5) Data Processing*. Calculate the average and standard deviation of the OD values of miR-1301 and the control pcDNA3, and draw a bar graph.

#### 3.3.3. CCK-8 Method Used to Detect the Proliferation of YD-38 Cells

In order to explore the difference in the migration ability of squamous cell carcinoma YD-38 cells, the cell scratch test was used to detect the cell migration ability. Using the in vitro cell healing experimental model to observe the migration ability of human squamous cell carcinoma YD-38 cells, the measurement time is 24 h, 48 h, and 72 h after transfection.

#### 3.3.4. Determination of YD-38 Cell Migration Level

After transfection, the measurement time was 24 h, 48 h, and 72 h, and monolayer cells were prepared.

Digest and count logarithmic growth phase squamous cell carcinoma YD-38 cells, add 500 *μ*L cell suspension (6 × 10^4^ cells) to a 24-well plate, 3 replicate wells in each group, and incubate for 24 h. The cells used in the migration test were placed in an incubator for 24 hours, and then the scratch test was performed. To detect the influence of miR-1301 on cell migration ability, the cells in the experiment were placed in an incubator for 24 hours and then transfected. The number of squamous cell carcinoma YD-38 cells inoculated and the volume of transfection reagent were converted according to the ratio of the bottom area of the culture plate. The paper used scratch experiments to conduct cell culture experiments to detect their migration ability, which partly mimics the process of cell migration in vivo. It has a low price and is easy to operate. It is also important that the cell peripheral environment is simple and easy to control. Compatible with microscope systems including live-cell imaging, it can be used to analyze cell to cell interactions. Here, we analyzed the culture duration of cells in 10 incubators, 48 h and 72 h to examine the effect of miR-1301 cell migration by 24 h, respectively.

The next day, use tweezers to take out the Transwell cell, first pour out the culture medium in the upper cell, fix it in the fixative (methanol: glacial acetic acid = 3 : 1) for 30 minutes, wash the cell three times with PBS, wipe the upper cell with a cotton swab, and then use stain with 0.1% crystal violet staining solution for 20 minutes. Scratch experiment was performed 48 h after transfection. Use a 100 *μ*l pipette tip to make a mark of “one” on the cells, wash 3 times with PBS, add culture medium, parallel three samples, observe and take pictures under an inverted phase-contrast microscope, incubate in the incubator for 24 hours, suck off the culture solution, PBS wash 3 times, calculate the average distance and standard deviation of cell migration, and draw a histogram.

#### 3.3.5. Western Blot Measures the Expression of PI3K, p-AKT, and AKT Protein in YD-38 Cells

1. Extraction of total cell protein: 48 h after transfection, aspirate the original medium, rinse with PBS 3 times, add 300 *μ*L of RIPA lysis buffer containing protease inhibitors, and shake for 30 min in an ice bath. Finally, centrifuge at 14000 rpm for 15 min. The resulting supernatant is the protein sample.
2. Detection of protein concentration: take 2 *μ*L of protein page and use it with ND2000 micronucleic acid protein detector for detection and recording. Carry out the following experiment or store at −80°C.
3. Protein sample denaturation: adjust the concentration of each histone sample in the experiment to be consistent, and then mix and configure according to the ratio of 5 × buffer to protein volume ratio of 1 : 4; pipetting several times, next, it can be observed that the most suitable storage temperature is −20°C according to its residence time in boiling water.
4. Preparation of SDS-PAGE gel: according to the gel kit instructions, first prepare 10% 15 ml separation gel, mix well, quickly fill the gel with a pipette, fill the two plates with the same volume, and then inject saturation on the separation gel solution n-butanol; after standing at room temperature for 30 minutes, suck up the n-butanol with a syringe, add 1 ml ddH2O, tilt the rubber plate to wash it back and forth, pour off the water, then use filter paper to absorb the rubber surface, then prepare 6 ml concentrated glue, and fill the glue quickly, Immediately insert the corresponding tooth comb, and leave it at room temperature for 30 minutes to agglomerate the concentrated glue.
5. Electrophoresis: unplug the tooth comb, pour sufficient Tris-glycine buffer into the electrophoresis tank, group samples according to the experiment, 30 *μ*L per well, set the voltage to 80 V (current about 40 mA) for 30 min at the beginning, and wait for it to be mixed with bromine. When the protein sample of the phenol blue stain reaches the separation gel layer, the voltage is increased to 100 V, and when it reaches the separation gel bottom layer, the power is turned off.
6. Transfer film: take out the gel glass plate, pry the glass plate from the corner with tweezers, then gently separate the glue from the glass plate with tweezers, cut off the concentrated glue, and then follow the negative electrode-sponge-3 layers of filter paper-gel Glue-methanol activated PVDF membrane-filter paper 3 layers-positive electrode order, be careful not to have bubbles between the layers during the operation, prepare to transfer the membrane, put the wet transfer instrument in ice water, and turn on the power supply and constant current 350 mA, 90 min. When finished, turn off the power.
7. Development and the result of the analysis: after 2 h, wash 4 times with 1 × TBST, 5 min each time, prepare ECL color developing solution at the same time, mix AB solution according to the volume ratio of 1 : 1, and avoid light. The PVDF film reacts in the developer solution for about 1 min, and then the gel imager is used for imaging. Using ImageJ software to analyze, compare the target protein caspase3 band with the housekeeping gene protein band and the result is the relative expression level of the target protein caspase3. After transfection, the measurement time is 24 h, 48 h, and 72 h.

## 4. Under Deep Learning Medical Images, Exploring the Experimental Research and Analysis of miR-1301 Inhibiting the Proliferation and Migration of Squamous Cell Carcinoma YD-38 Cells through the PI3K/AKT Pathway

### 4.1. mRNA Expression of miR-1301 In HGF-1 and YD-38 Cells

In this paper, HGF-1 and YD-38 cells are routinely cultured in vitro. When the cells enter the logarithmic growth phase, the original culture medium is discarded. The first group adds miR-1301 mimics and the other group adds miR-1301 blanks. Readd a small amount of serum-free culture medium and continue to culture in the incubator. After collecting the supernatant, the mRNA expression level was detected by the Western blot method. Each experiment was repeated three times as shown in Figure 1.

As shown in Figure 1, the addition of miR-1301 mimic compared with the miR blank group shows that the mRNA content in the cells with miR-1301 mimic added is different from that in the cells without miR-1301 mimic. The miR-1301 mimic group is slightly higher than the miR-1301 blank group, with statistical significance (*P* < 0.05).

### 4.2. YD-38 Cell Proliferation Level

The YD-38 cells were transfected with miR-1301 mimics and the control miR blank group, and the growth of YD-38 cells after transfection with different plasmids was detected experimentally. The experimental results are shown in Figure 2.

The experimental results are shown in Figure 2. The results indicate that in these two sets of experiments, the absorbance measured at 450 nm of YD-38 cells in the miR-1301 mimic group is lower than that of the control group. It can be seen that the overexpression of the miR-1301 mimic group inhibits YD-38 cell proliferation ability; the difference was statistically significant (*P* < 0.05).

### 4.3. Determination of YD-38 Cell Migration Level

In order to explore whether miR mimics will affect the migration ability of YD-38 cells, this paper uses a cell scratch test to detect cell migration ability. Using the in vitro cell healing experimental model for reference, the effect of miR mimics on the migration ability of YD-38 cells was observed. The experimental results are shown in Figure 3.

The results showed that the migration distance of YD-38 cells in the miR mimic group was 2.2 ± 0.31 times that of the YD-38 cells in the miR blank group by observing the two groups of cells. It is suggested that the miR blank group has a stronger ability to inhibit the migration of YD-38 cells compared with the miR mimic group. As shown in Figure 3, the migration level of YD-38 cells in the miR simulation group decreased within 72 hours from 42% to 26%, and in the miR blank group, YD-38 cells decreased from 38% to 16%, which was significantly faster in the miR simulation group, indicating that the mimic significantly enhanced YD-38 cells.

### 4.4. YD-38 Cell PI3K, p-AKT, and AKT Protein Expression

The scanned images of the Western blotting experiment were quantitatively analyzed in the gel image analysis software. The relative expression levels of PI3K, p-AKT, and AKT proteins (PI3K, p-AKT, and AKT) are expressed in terms of relative gray values. The experimental results are shown in Figure 4.

As shown in the Western blot of the experimental results in Figure 4, it can be seen that after treating YD-38 cells for different times in the miR mimic group and the miR blank group, compared with the 24 h group, the miR mimic group treated for 24, 48, and 72 h, the expression of AKT was significantly downregulated, and the phosphorylation level of AKT was also significantly reduced (*P* < 0.05).

## 5. Conclusion

miR-1301 is low expressed in oral squamous cell carcinoma YD-38 cells and inhibits its proliferation and migration. To a certain extent, the experiment may be related to the pathway activity of cells by selecting the control group and blank group simulated by miR, as well as pathway inhibitors, and they can be combined therapy at the same time. After 72 hours of treatment, the results of the scratch test and the in vitro migration and invasion test of the Transwell chamber showed that, in contrast, YD-38 cells treated with the simulant can be seen to have lower migration and reproduction capacity, which is very good indicating that ERS promoted the migration and proliferation of YD-38 cells, indicating that miR-1301 inhibits the migration and proliferation of cells by blocking the PI3K/AKT pathway. This result suggests that miR-1301 may block the migration and proliferation of YD-38 cells through the PI3K/AKT pathway.

## Figures and Tables

**Figure 1:** mRNA expression of miR-1301 in HGF-1 and YD-38 cells. ^*∗∗*^*P* < 0.01, compared with miR blank group.

**Figure 2:** YD-38 cell proliferation level. ^*∗*^*P* < 0.05 and ^*∗∗*^*P* < 0.01, compared with miR blank group.

**Figure 3:** Measurement of YD-38 cell migration level. ^*∗*^*P* < 0.05 and ^*∗∗*^*P* < 0.01, compared with miR blank group.

**Figure 4:** The expression of PI3K, p-AKT, and AKT protein in YD-38 cells. ^*∗∗*^*P* < 0.01, compared with the miR blank group.

## Data Availability

Data cannot be made available because no analytical permission was obtained from the data provider due to trade confidentiality.
